The article "Automated System for Identifying COVID-19 Infections in Computed Tomography Images Using Deep Learning Models" was retracted in 2023. Reasons: signs of a paper mill; suspected computer-generated content; unreliable results or conclusions; concerns about the data.

# Automated System for Identifying COVID-19 Infections in Computed Tomography Images Using Deep Learning Models

**DOI:** 10.1155/2022/5329014

**Published:** 2022-03-30

**Authors:** Karrar Hameed Abdulkareem, Salama A. Mostafa, Zainab N. Al-Qudsy, Mazin Abed Mohammed, Alaa S. Al-Waisy, Seifedine Kadry, Jinseok Lee, Yunyoung Nam

**Affiliations:** ^1^College of Agriculture, Al-Muthanna University, Samawah 66001, Iraq; ^2^Faculty of Computer Science and Information Technology, Universiti Tun Hussein Onn Malaysia, 86400 Batu Pahat, Johor, Malaysia; ^3^Computer Sciences Department, Baghdad College of Economic Sciences University, Baghdad, Iraq; ^4^College of Computer Science and Information Technology, University of Anbar, 11 Ramadi, Anbar, Iraq; ^5^Communications Engineering Techniques Department Information Technology Collage, Imam Ja'afar Al-Sadiq University, Baghdad, Iraq; ^6^Faculty of Applied Computing and Technology, Noroff University College, Kristiansand, Norway; ^7^Department of Biomedical Engineering, College of Electronics and Information, Kyung Hee University, Yongin-si, Gyeonggi-do 17104, Republic of Korea; ^8^Department of Computer Science and Engineering, Soonchunhyang University, Asan 31538, Republic of Korea

## Abstract

Coronavirus disease 2019 (COVID-19) is a novel disease that affects healthcare on a global scale and cannot be ignored because of its high fatality rate. Computed tomography (CT) images are presently being employed to assist doctors in detecting COVID-19 in its early stages. In several scenarios, a combination of epidemiological criteria (contact during the incubation period), the existence of clinical symptoms, laboratory tests (nucleic acid amplification tests), and clinical imaging-based tests are used to diagnose COVID-19. This method can miss patients and cause more complications. Deep learning is one of the techniques that has been proven to be prominent and reliable in several diagnostic domains involving medical imaging. This study utilizes a convolutional neural network (CNN), stacked autoencoder, and deep neural network to develop a COVID-19 diagnostic system. In this system, classification undergoes some modification before applying the three CT image techniques to determine normal and COVID-19 cases. A large-scale and challenging CT image dataset was used in the training process of the employed deep learning model and reporting their final performance. Experimental outcomes show that the highest accuracy rate was achieved using the CNN model with an accuracy of 88.30%, a sensitivity of 87.65%, and a specificity of 87.97%. Furthermore, the proposed system has outperformed the current existing state-of-the-art models in detecting the COVID-19 virus using CT images.

The article "Automated System for Identifying COVID-19 Infections in Computed Tomography Images Using Deep Learning Models" was retracted in 2023. Reasons: signs of a paper mill; suspected computer-generated content; unreliable results or conclusions; concerns about the data.

## 1. Introduction

Coronavirus disease 2019 (COVID-19) is a novel disease that rapidly spreads and affects the daily patterns of millions of people in the world. [1]. The infection causes pulmonary complications, such as severe pneumonia, which leads to death in several cases [1, 2]. The possible containment of this virus requires quick detection to ensure that the exposed person can be isolated as quickly as possible to mitigate the spread of the disease because it is highly contagious. Reverse transcription-polymerase chain reaction (RT-PCR) [1] is the standard method used to detect COVID-19; in this method, sputum or nasopharyngeal swab is tested for the presence of the viral RNA. RT-PCR has the following limitations: the long time required to produce results, limited or lack of test materials in medical centers and hospitals [2], and relatively low sensitivity; this condition is not conducive to the main objective of detection of rapid positive samples for immediate isolation [3]. The utilization of medical images, such as chest X-ray images or computed tomography (CT) scans, can be an alternative solution for fast screening [4]. An early-stage identification of COVID-19 via imaging would allow rapid patient isolation and thus would reduce the spread of the disease [1]. However, physicians are trying hard to contain this disease. Thus, artificial intelligence- (AI-) based decision support tools should be developed to identify and use the image at the lung level in segmenting the infection [2]. AI, such as machine and deep neural network (DNN) techniques [5], has been increasingly used in recent years as the main tool to find solutions to diverse difficulties, such as object detection [6–8], image classification [9], and speech recognition [10]. In image processing [11], a convolutional neural network (CNN) has specifically produced outstanding results [12]. Many studies have presented the influence and strength of these techniques in image segmentation [13]. Image classification [14] and image segmentation [13] for medical imaging has also produced very good results using CNN architectures [15].

The most effective technique for detecting lung COVID-19 is CT because of its 3D image-forming capability of the chest, which enables it to produce lung pathology in greater resolution. Computer processing of a CT image is a popularly used technique in aiding clinical lung COVID-19 diagnostics. The use of a computer-supported identification process for lung COVID-19 can be divided into two: a detection system and an identification approach (usually abbreviated as CAD). The CAD approach categorizes the previously identified candidate lung COVID-19 as normal or nonnormal COVID-19 cases (i.e., normal anatomic structures). The detected lung inflammation is classified as normal or nonnormal as COVID-19 by the CAD approach [16]. The CAD can differentiate the lung inflammation as normal or nonnormal COVID-19 case by utilizing efficient features, such as shape, texture, and growth rates because a probability has a close relationship to shape, geometric size, and appearance in COVID-19. Thus, the precise diagnostic, speed, and automation levels are measurable terms that can present the achievement of a specific CAD approach [17].

The article "Automated System for Identifying COVID-19 Infections in Computed Tomography Images Using Deep Learning Models" was retracted in 2023. Reasons: signs of a paper mill; suspected computer-generated content; unreliable results or conclusions; concerns about the data.

Deep learning enhances the accuracy of the computerized process and assessment of CT image segmentation and identification and accelerates the critical task. The problem associated with lung inflammation classification into normal or nonnormal COVID-19 cases is considered in this study. However, several existing CT scan datasets for COVID-19 comprise hundreds of CT images and fall short of the demand [18]. Several available COVID-19 datasets also lack fine-grained pixel-level annotations; they also provide only the patient-level labels (i.e., class labels), which indicate whether the person is infected or otherwise [19, 20]. DNN, CNN, and stacked autoencoder (SAE) are proposed to implement COVID-19 identification. The research can be utilized directly as input to limit the difficult data reconstruction process during feature extraction and classification. This study constructs a large-scale CT scan dataset for COVID-19 that comprises pixel-level annotations to alleviate the limitations presented earlier. Then, we propose a CT diagnosis system for COVID-19 classification to provide explainable diagnostic results to medical staff battling COVID-19. We specifically use the gathered COVID-19 CT dataset from hundreds of COVID-19 cases containing thousands of CT images to train the employed deep learning models for better diagnosis performance. The proposed diagnosis method first identifies the suspected patients of COVID-19 using a classification model based on lung CT images. Then, the system provides the diagnosis explanations by applying activation mapping techniques. The proposed system can find the locations and areas of the lung radiography using fine-grained image techniques. Our method extensively accelerates and simplifies the diagnosis procedure for radiologists related medical personnel by providing them with explainable classification results. Accordingly, our contribution is summed up in three main points as follows:

- We showed that the proposed classification techniques and their implemented models can effectively improve the performance of COVID-19 diagnosis by using limited computational resources, few parameters, and only 746 chest CT scan samples
- We proposed a new COVID-19 diagnostic model to perform explainable detection and precise COVID-19 case classification and show significant improvement over previous systems
- The proposed CNN, DNN, and SAE use CT scans as a direct input to limit the complexity involved with data reconstruction during the deep learning and classification processes

This paper is structured in five sections, and the following section evaluates the previous studies, while Section 3 contains the presentation of the materials and methods for classifying lung CT images.  Section 4 shows the produced experimental outcomes, and Section 5 elaborates the conclusion of our study.

The article "Automated System for Identifying COVID-19 Infections in Computed Tomography Images Using Deep Learning Models" was retracted in 2023. Reasons: signs of a paper mill; suspected computer-generated content; unreliable results or conclusions; concerns about the data.

## 2. Related Work

The complexity in the diagnostic of inflammatory and infectious lung disease using visual examination is still a challenge in developing an automated system for lung CT scan classification. The large number of patients requiring diagnosis is a source of errors for an acceptable standard as visual examination. Wang et al. [16] proposed a system to offer a clinical identification of the pathogenic examination using CNN-based automated technique in identifying distinct COVID-19 features. The dataset contained 217 cases and produced an accuracy of 82.9%. A fully automated framework was proposed by Li et al. [21], and it utilized a CNN for extracting the best features in detecting COVID-19 and distinguishing it from the healthy case and pneumonia infection. The used dataset contained 400 CT scans and produced an overall accuracy of 96% in detecting COVID-19 cases. Xu et al. [22] proposed an automatic screening approach utilizing deep learning methods to distinguish CT samples detected with influenza-A viral pneumonia or COVID-19 from the sample of patients who had healthy lungs. The dataset contained 618 lung CT scans and produced an overall classification accuracy of 86.7%, as revealed by the experimental result. Song et al. [23] improved an automatic deep learning identification approach to aid medical personnel in detecting and recognizing patients infected by COVID-19. The gathered dataset contained CT scans of 86 healthy, 88 COVID-19, and 100 bacterial pneumonia samples. The proposed deep learning model could detect and classify bacterial pneumonia and COVID-19-infected samples with an accuracy of 95%. Hasan et al. [24] presented identification COVID-19 among COVID-19, healthy, and pneumonia CT lung scans using the integration of Q-deformed entropy handcrafted features and deep learning of extracted features. Preprocessing was utilized to limit the intensity difference influence amid CT cases in this study. In isolating the background of the lung CT scan, histogram thresholding was applied. Feature extraction was conducted on every lung CT scan using a Q-deformed entropy and deep learning methods. The long short-term memory (LSTM) type of neural network was employed to classify the extracted features. The combination of all features extracted meaningfully resulted in better execution of the LSTM network in accurately discriminating among COVID-19, healthy, and pneumonia samples.

The article "Automated System for Identifying COVID-19 Infections in Computed Tomography Images Using Deep Learning Models" was retracted in 2023. Reasons: signs of a paper mill; suspected computer-generated content; unreliable results or conclusions; concerns about the data.

Feature extraction complexity is one of some limitations in present classification models. Feature extraction algorithms play a vital role in gathering the significant variations in the spatial scattering of image pixels. The powerful discriminative capability of AI technologies, especially deep CNNs, is improving medical imaging solutions. However, deep learning algorithms, including CNNs need to be trained on large-scale datasets to show their capability. The majority of presently available CT scan datasets for COVID-19 [25, 26] comprise hundreds of CT images from tens of cases, which fall short of the requirement. Lack of fine-grained pixel-level annotations and provision of patient-level labels (i.e., class labels) that indicate whether the person is infected in the majority of the currently available COVID-19 datasets makes CNN models trained. Despite the establishment of several diagnosis systems for testing suspected COVID-19 cases by CT scan [27], most of them exhibit two constraints: (1) they are not suitably robust for versatile COVID-19 infections because they are trained on small-scale datasets; (2) they lack explainable transparency in assisting doctors during medical diagnosis because classification is performed on the basis of black-box CNNs.

The lung CT scan classification models in existing systems depend on deep learning methods to extract the best features. The classification performance between healthy and COVID-19 cases will improve further as a result of deep learning features. Proposing an efficient COVID-19, healthy, and COVID-19 lung classification in CT images applying the deep learning models is the motivation for this study. CNN, DNN, and SAE provide the means of developing a COVID-19 diagnosis method that can perform supervised learning and produce accurate detection.

## 3. Materials and Methods

There is a significant require for speedy testing and diagnostic of patients amid the COVID-19 widespread. Lung CT is an images methodology that is widely accessible and cost-effective and can analyze and diagnose intense respiratory trouble disorder in patients with COVID-19. It can be utilized to discover imperative features within the medical samples that present all the clinician information that can be used to diagnose and monitor the COVID patents. With the usage of versatile ultrasound transducers, lung CT samples can be effortlessly obtained. In any case, the CT image is frequently of destitute quality. It frequently needs a specialist clinician elucidation, which may be highly subjective and time-consuming. The main goal of this work is to develop a new COVID-19 identification framework proposed to automatically distinguish between COVID-19 infected subjects and healthy one via CT images using different deep learning methods.

The article "Automated System for Identifying COVID-19 Infections in Computed Tomography Images Using Deep Learning Models" was retracted in 2023. Reasons: signs of a paper mill; suspected computer-generated content; unreliable results or conclusions; concerns about the data.

### 3.1. CT Image Dataset

The dataset consists of 746 COVID-19 patient cases with their CT scan images and full clinical description (e.g., 349 images with confirmed COVID-19 infection, while 397 CT scans belong to individuals with a good health condition and no diagnosed pneumonia diseases) [25]. Free public radiology resources, including datasets, reference studies, case studies, and CT images, are provided on many international radiology websites, such as medRxiv and bioRxiv. The first COVID-19 dataset used in our study is obtained from medRxiv and bioRxiv for the period from January 19, 2020, to March 25, 2020. An example of chest CT scans for patients having COVID-19 is shown in Figure 1.

### 3.2. Automated COVID-19 Classification Methodology

This research aims to enhance the process of COVID-19 identification and diagnosis by minimizing the diagnostic error rate associated with human error in reading chest CT scans. In addition, it aims to help medical practitioners conduct fast identification to distinguish among the patients with confirmed COVID-19 infection, other pneumonia infections, and healthy people. The proposed system can be divided into three major phases: preprocessing of CT images, extraction of dominant features, and classification of selected features by DNN, CNN, and SAE classifiers to make the final decision.  Figure 2 illustrates the components of the proposed COVID-19 identification.

#### 3.2.1. CT Lung Preprocessing Stage

The quality of the image scan depends on the accuracy of the metrics, intensity, and variations of the reconstructed and consecutive slices of CT scan [28]. Normalization of the intensity through extracting deep features can help minimize the CT slice variations, enhance the classifier's performance, and accelerate the training process. This process also identifies lung boundaries to recognize the area of thoracic tissue surrounding the lung, which is represented as many unimportant pixels [29]. We use the histogram thresholding method that isolates each individual CT with intensity values larger than a set cut-off value from the CT lung background pixels. Then, the morphological dilation operation was applied to fill the gaps that appear in the sliced image. Any deficiencies found can be removed by connecting small objects. As a result, the shades of zeros and ones are applied to extract the more interesting area of the lung. Ones represent the lung area, and the background is represented by zeros [22]. Algorithm 1 describes the pseudocode of the steps of the chest CT scan. A sample of the segmented CT lung is illustrated in Figure 3.

The article "Automated System for Identifying COVID-19 Infections in Computed Tomography Images Using Deep Learning Models" was retracted in 2023. Reasons: signs of a paper mill; suspected computer-generated content; unreliable results or conclusions; concerns about the data.

#### 3.2.2. Deep Learning for Feature Extraction

The use of handcrafted features as input to the classifier with expert guidance may affect its performance. However, many deep learning techniques perform more successfully in extracting features, particularly in the computer vision domain. They also show efficiency in improving the accuracies of classification. In this study, the CNN technique is used to extract features efficiently. CNN is one of the successful classification methods in the computer vision domain. CNN is an improved version of the classical neural network by introducing new layers (convolutional, pooling, and fully connected) [30]. The convolutional layers consist of a number of trainable convolutional filters.

The filters change the entire input size to be specific amount known as stride(s) to yield integer dimensions of output size [31]. As a result of this process, the spatial dimensions of input size are considerably reduced after the convolutional layer. The original input size with a low number of features needs to be minimized by zero-filling each input to be assigned with zero value. In the feature maps, all negative values are turned to zeros via the rectified linear unit (ReLU) layer to maximize the feature maps nonlinearly. Thereafter, the pooling layers divide the feature maps into small nonoverlapped partitions to minimize the data dimensionality. For this purpose, the pooling layer has been supported by the max-pooling function in this research. A batch normalization layer performs normalization of the features to accelerate the training process. The fully connected layer is considered the most significant layer in CNN. The normalized feature map is inserted into this layer, and this layer acts as a classifier to yield the final results and label probabilities. Although CNN is a powerful method as a classifier, it has a disadvantage in terms of requiring intensive parameter tuning. As a result, fewer convolution layers are used to reduce the complexity of CNN architecture and thus the parameter tuning process. CNN aims to extract highly significant features for a particular task. The network architecture, the number of convolutional layers, the filters size, and the CT partitions inserted into the network are major factors that affect the classification process. Therefore, they should be given more attention when applying CNN. In our study, the CT slice dimensions are set to (256 × 256) pixels to reduce computation complexity. For a given CT partition, the size of the convolutional layer and the number of zero-filling are determined via the following equations:

(1) $$\begin{array}{c} {\text{Conv}}_{\text{width}}=\frac{CT{\text{Slice}}_{\text{width}}-Cf_{\text{width}}+\left(2\times ZP_{\text{width}}\right)}{S_{\text{width}}}+1,\\ {\text{Conv}}_{\text{height}}=\frac{CT{\text{Slice}}_{\text{height}}-Cf_{\text{height}}+\left(2\times ZP_{\text{height}}\right)}{S_{\text{height}}}+1,\\ ZP_{E}=\frac{Cf_{\text{width}}-1}{2},\\ ZP_{\text{height}}=\frac{Cf_{\text{height}}-1}{2}. \end{array}$$

The article "Automated System for Identifying COVID-19 Infections in Computed Tomography Images Using Deep Learning Models" was retracted in 2023. Reasons: signs of a paper mill; suspected computer-generated content; unreliable results or conclusions; concerns about the data.

#### 3.2.3. The Convolutional Neural Network (CNN)

CNN is a neural network based on a multilayer approach. It consists of a set of convolution and fully connected layers; the latter acts as the standard layer of the neural network. The idea of CNN can be traced back to the 1960s [32]. It is based on three concepts: local perception, sharing of weights, and time or space sampling. Local perception is an efficient detection method that is currently attracting attention. This method mainly detects the local aspect of data to extract the basic features for the visual object in a picture, such as an angle or arc of an animal [15]. The advantage of CNN is the requirement of a few parameters compared with the number of hidden units for fully connected networks. CNN consists of two layers: the convolution and pool layers that collaborate [33]. It may affect a specific position of the features and make a confusion of uninterested feature location to focus on other relative positions of features. The pooling layer function relies on mean pooling and max-pooling operations. Mean pooling operation computes the neighborhood average of feature points, while max-pooling operation computes the maximum of feature points for the neighborhood. The size limitation of the neighborhood may cause a feature extraction error. The reason is that the mean deviation is due to errors of the estimated parameter and variance in the convolution layer. Estimated variance error can be decreased by mean pooling operation by preserving image background information. Estimated parameter error can be decreased by max-pooling operation by preserving image texture information.

The CNN architecture is illustrated in Figure 4. The CNN architecture comprises multiple layers. Every layer comprises multiple maps. Every map comprises numerous neural units. For the same map, neural elements share the weight of the convolution kernel. Every convolution kernel is shown as a feature. The edge of image features can be accessed. Additional CNN details are represented in Table 1. Image data, which are represented as input data, have high control of the deformation. The convolution kernel and parameter size generate the multiscale image feature convolution. The distinct angles of information are created in the space of feature.

The article "Automated System for Identifying COVID-19 Infections in Computed Tomography Images Using Deep Learning Models" was retracted in 2023. Reasons: signs of a paper mill; suspected computer-generated content; unreliable results or conclusions; concerns about the data.

#### 3.2.4. The Deep Neural Network (DNN)

A DNN is a basic neural network with more hidden nodes. An intensive computation of the input is conducted in the neural network because of the nonlinear transformation from each hidden layer to the output layer [34]. However, DNN is more efficient than the superficial network. As for the linearity of the activation function, each hidden layer should be represented as the nonlinear function *f*(*x*). This condition is opposite to the individual hidden layer in the neural network, given that the hidden layer depth has no ability to improve the expression. The aspect of various sizes of the lung nodes is extracted from different network layers in the DNN processing phase. DNN has some issues with respect to problems associated with the local boundary and gradient spread. The original image is fed as the input in the training process to preserve more image information.

The DNN architecture comprises the input, hidden, and output layers. All these layers are interconnected to one another. DNN has no convolution layer. Training and label images are fed to the DNN. In the initial training, the random weight is assigned to every layer using Gauss distribution with bias equals to zero. Forward propagation is used for output calculation, while backpropagation is used for parameter updating. The depth structure of the neural network is illustrated in Figure 5. Additional neural network details are shown in Table 2. The DNN requires sorting out some issues related to its parameters, including the tuning of parameters, the growth of data size, and normalization [35, 36].

#### 3.2.5. The Stacked Autoencoder (SAE)

An SAE is an unsupervised learning algorithm having a multilayer neural network with SAE [37]. It consists of input, hidden, and output layers. The SAE architecture is shown in Figure 6. The input and output layers have the same number of neurons, while the hidden layer has less number of neurons. The SAE is composed of two phases: the coding and decoding phases. Mapping from the hidden and input layers occurs in the coding phase. Meanwhile, mapping the hidden layer to the output layer occurs in the decoding phase.

The article "Automated System for Identifying COVID-19 Infections in Computed Tomography Images Using Deep Learning Models" was retracted in 2023. Reasons: signs of a paper mill; suspected computer-generated content; unreliable results or conclusions; concerns about the data.

This research uses a combination of multiple autoencoders and softmax as a classification method to build an SAE network. The SAE network has several hidden layers and softmax as a final layer [38]. Sparse autoencoder, which is a variant of autoencoder, was introduced in [39]. SAE has very few active neurons. Masci et al. [40] proposed a convolutional autoencoder that trains high-dimensional image data. However, this convolution structure has difficulty in training the autoencoder in a convolutional way because of the high computational load and complex architecture [41].

The architecture of the SAE neural network is shown in Figure 7. The hidden layer includes an individual hidden layer of the scattered autoencoder. Identification of pulmonary nodes is considered an image classification problem. Each scattered autoencoder removes the decoded layer by the end of the training process. Then, the encoding process is started to train the next output of SAE.

#### 3.2.6. Loss Functions for Neural Network

In the loss function, the last element is used to restrain overfitting for the training procedure, and the aggregate of weights is distributed by *n* multiplied by 2. Dropout is also used to restrain overfitting. Random neurons are protected prior to backpropagation. Thus, updating parameters of shaded neurons is not allowed. DNN requires a large number of data as input for the neural network, and this condition requires large memory storage. Min_batch is used in the backpropagation to accelerate the updating process of parameters for solving the aforementioned issue. The loss function is formulated and explained as follows:

(2) $$\begin{array}{c} C\left(w,b\right)\equiv \frac{1}{2n}\sum_{x}{\left\|y\left(x\right)-a\right\|}^{2}+\frac{1}{2n}\lambda \sum_{w}w^{2}. \end{array}$$

Here, C represents the total function, *w* represents the weight, *b* represents the bias, *n* represents the training dataset instance numbers, and *x* is an input parameter that represents the values of the image pixel and output. The backpropagation method is adopted in DNN to update the *b* weight wand for enhancing accuracy by reducing the difference between the expected and actual values.

The leaky ReLU represents a neural network's activation function that helps improve the nonlinear modeling ability. The ReLU activation function is formulated as follows:

(3) $$\begin{array}{c} y=\left\{\begin{array}{cc} x, & \text{if}x\geq 0,\\ 0, & \text{if}x<0, \end{array}\right. \end{array}$$

where *x* represents the weighted priority multiplication result and weight wand added to the *y* element to obtain the activation function output. The ReLU derivative can be 0 if *x* < 0; otherwise, it can be 1. ReLU can remove the gradient sigmoid activation function problem. However, the phenomenon of neuronal death can occur as the updating weight is stopped because of the continuous updating in the training process. In this situation, the ReLU output can be more than zero, which means the neural network output is offset.

The article "Automated System for Identifying COVID-19 Infections in Computed Tomography Images Using Deep Learning Models" was retracted in 2023. Reasons: signs of a paper mill; suspected computer-generated content; unreliable results or conclusions; concerns about the data.

This problem can be solved by applying the leaky ReLU method. This method is an activation function that can be represented as follows:

(4) $$\begin{array}{c} y=\left\{\begin{array}{cc} x & \text{if}x\geq 0,\\ ax & \text{if}x<0, \end{array}\right. \end{array}$$

where a is set to 0.1. Notably, a is a fixed value in leaky ReLU, while a is not fixed in the ReLU.

#### 3.2.7. Data Augmentation

Data augmentation refers to the differences in sizes of lung patterns. The size of lung patterns is regularly set to 28 × 28 to extract the aspects of the lung patterns, including the size and texture. Binary processing is used to obtain lung pattern images [42]. They can be approximately outlined. Subsequently, the lung pattern value is preserved as pixels in the advanced image. Finally, any noise perturbation that surrounds the lung patterns is removed [43]. The neural network training entails a large number of positive and negative samples. In this study, we first process the images' translation, flip, and rotation. Then, we insert them as the input of the neural network to maximize the size of the sample data. The large size of the sample data can positively affect the performance of the neural network in terms of enhancing the training process, improving the accuracy of testing, decreasing the loss function, and increasing the efficacy of the neural network.

## 4. Experimental Results and Discussion

This section presents the experiment configuration settings and the outcomes of the proposed systems based on the classification of the CT scan images. Two main subsections are presented as follows:

### 4.1. Experiment Settings

Caffe, a deep learning model based on expressiveness, modularity, and speed, is used in this research. A total of 746 CT scans are used, which comprise 349 CT scans for COVID-19 hospitalized individuals' CT scans for infected pneumonia patients, and 397 CT scans for healthy persons with no apparent chest infection. The first website publicly offers reference documents, radiology images, and patients' cases. The latter contains open access datasets with a wide archive of medical images with public viewing. The second website is a partnership on radiology. A total of 20% of the training data, which comprise approximately 448 images, are utilized for cross-validation. The same set of data applies to the three distinct architectures of the network.

The article "Automated System for Identifying COVID-19 Infections in Computed Tomography Images Using Deep Learning Models" was retracted in 2023. Reasons: signs of a paper mill; suspected computer-generated content; unreliable results or conclusions; concerns about the data.

The learning rate of the CNN is set to 0.02, and the batch size is set to 24 during network training to obtain the best results. The process of convolution and sampling is performed twice in the network. The kernel size is 6, and two layers of convolution are considered and consist of 36 filters. The pooling layer has a kernel size of two. The purpose of a dropout layer is being used to avoid overfitting. At least a softmax function with two fully connected layers is considered. The DNN contains a completely connected layer.

The 2D data input of 24 × 24 mapped into 576 × 1 is presented as an input image in the first layer. An entirely connected layer of 304 × 1 is used in the second layer. The third layer is fully connected to 256 × 1. A dropout layer will be considered after the third layer, which includes a parameter of 0.5. Units will also be hidden in 30%. The fully connected layer is the fourth layer of 128 × 1 with ReLU as an activation function. The SAE structure also consists of a completely connected layer. The input and output neurons of the automotive encoder are the same. Thus, the autoencoder is the same as

(5) $$\begin{array}{c} H_{w,b}\left(x\right)=x. \end{array}$$

Here, *w* and *b* are the crankiness and weight, respectively; *x* is the input factor. The neural networks correspond to the input image coding. The self-encoder creates the hidden layer, and it is primarily utilized in the identification process. This way cancels the self-encoder decoding portion. The coding factor of the SAE is utilized during training. The encoder creates a stack encoding component to add a confident number of training courses to the identification of the initializing neural network. The artifact characteristics are not evident after the encoder the image edge is formed. However, this condition triggers some reduction in classification accuracy.  Table 3 offers information on the SAE.

### 4.2. COVID-19 Classification Results

This section presents the classification of CT COVID-19 and normal cases. The classification results are based on the experiment outcomes of three deep learning models: CNN, DNN, and SAE. Accuracy, sensitivity, and specificity are used as evaluation indicators for the performance of the three mentioned models. The classification results of the three models are presented in Table 4.

The results show that the CNN has a sensitivity of 87.65%, a specificity ratio of 87.97%, and an accuracy of 88.30%. The accuracy, sensitivity, and specificity of DNN are 86.23%, 84.41%, and 86.77%, respectively. The good result is due to the fact that the operation of the convolution layer can be defined by the texture and shape of two distinct dimensions. A convolution kernel shares constraints throughout the procedure of convolution in diverse weights for diverse image features with a convolution kernel. Thus, the convolution operation is less than the fully connected operating conditions in terms of parameter number. The DNN has poor precision and sensitivity than the SAE. However, the former is better than the latter, given that it has a specificity ratio of 87.84%.

The article "Automated System for Identifying COVID-19 Infections in Computed Tomography Images Using Deep Learning Models" was retracted in 2023. Reasons: signs of a paper mill; suspected computer-generated content; unreliable results or conclusions; concerns about the data.

Better specificity provides a greater degree of detection of COVID-19 within a single set of data, and this feature can be more useful in slightly earlier diagnosis of pulmonary pathways. However, DNN increases the number of false-positive COVID-19 cases to a certain degree. The DNN and SAE are completely connected networks, but different generating methods are possible. In encoder training, SAE is generated by parsing; the DNN is generated directly from formation through the completely connected layer.

Unlike the previously published works that mainly depend on employing pretrained models in identifying the COIVD-19, we proposed to build a customized CNN model composed of two convulsion layers to reduce the number of hyperparameters and the model's complexity. On the contrary, the pretrained models such as ResNet and DenseNet have more complex architecture, which can present high computational load and execution time during training and validation processes. Furthermore, it is very difficult to change the main structure of the pretrained model by adding or removing some layers to find an optimal model's structure.

Certainly, the computing time of the model is an important problem in identifying the COVID-19 virus, where having a customized CNN model that required fewer CT images can significantly help the doctors in the early diagnosis of the COVID-19, especially when there is a very limited number of CT images with confirmed COVID-19 infection.

Finally, to compare the testing time required to produce the final decision per image of the proposed models and the current state-of-the-art works.  Table 5 lists the seconds' testing time per image to produce the final prediction results. From this table, one can see that the proposed models have outperformed all the current state-of-the-art works in terms of generating the final decision. Although Kassani et al. [44] achieved a faster testing time than the proposed DNN model, it has inferior results than the other two models (CNN and SAE model).

The evaluation scenario with other benchmarked studies is presented in Table 6. For a fair comparison, the experiments in this study are done on the basis of the same dataset and hyper tuning parameters. However, the experimental results and data of the CNN parameters can still be improved. CT lung COVID-19 image cases that include normal and COVID-19 samples are shown in Figure 8.

The article "Automated System for Identifying COVID-19 Infections in Computed Tomography Images Using Deep Learning Models" was retracted in 2023. Reasons: signs of a paper mill; suspected computer-generated content; unreliable results or conclusions; concerns about the data.

Table 6 shows that the benchmarking process that determines the efficiency and reliability is the most essential step in common medical image processing and diagnosis research. Benchmarking is achieved by utilizing the best recent prediction COVID-19 methods based on CT lung COVID-19 images based on deep learning approaches in the literature. As aforementioned, further evaluation of the present COVID-19 prediction system in CT lung COVID-19 images is made by benchmarking it with the best three studies from the CT lung COVID-19 image classification [42, 45, 46]. Table 6 summarizes the results after benchmarking. Common trends of performance and major measurements are classification accuracy rate (CAR), sensitivity (Sen.), and specificity (Spe.). The CNN scores an accuracy of 88.30%, a specificity ratio of 87.97%, and a sensitivity of 87.65%. The best performance in all benchmarked studies is observed with an accuracy of 86%, a sensitivity of 94%, and a specificity ratio of 79%. The proposed system presents an acceptable and significant sensitivity performance compared with the benchmarked studies with high sensitivity ratio. Nevertheless, the proposed system outperforms all the benchmarked studies in terms of accuracy and specificity performance.

## 5. Conclusion

This study aims to explore and extensively test three deep learning models. The prediction is compared for normal and COVID-19 cases by using chest CT images. Several preprocessing stages are applied to CT images. First, data segmentation is applied to isolate the region of interest from the CT image background. Second, a data augmentation technique is used to increase the volume of CT images. Accordingly, adequate input can be provided for the deep learning models for directly affecting the performance of classification. The test outcomes indicate that CNN achieves the ideal execution compared with the DNN and SAE. Moreover, the CNN is superior to other models in terms of performance with an accuracy of 88.30%, a sensitivity of 87.65%, and a specificity ratio of 87.97%. Neural network layers in this study are comparatively small due to the constraints of the datasets. The proposed approach is anticipated to increase the accuracy of the other database. Furthermore, deep learning approaches can be used to assist physicians in mitigating this newly spreading disease with CT images to identify and distinguish early COVID-19 patients, recognize and segment images in the medical field, and predict the results of treating them. We also show that too excellent sensitivity can be obtained from CT images, which can address the need for early-stage detection of infected persons to limit the progression of the virus. We will further validate the performance of our technique on a large dataset. The process can be generalized for the good implementation of CAD frameworks for future medical image processes. This study is limited to three models as diagnosis systems. However, additional deep learning models will be explored in the future.

The article "Automated System for Identifying COVID-19 Infections in Computed Tomography Images Using Deep Learning Models" was retracted in 2023. Reasons: signs of a paper mill; suspected computer-generated content; unreliable results or conclusions; concerns about the data.

## Figures and Tables

**Figure 1:** Positive cases for COVID-19 in CT scan images.

**Figure 2:** Proposed automated detection and classification of COVID-19 cases on CT images using deep learning models.

**Figure 3:** CT lung classification: (a) original CT lung case and (b) segmented CT lung.

**Figure 4:** CNN architecture.

**Figure 5:** DNN architecture.

**Figure 6:** Sparse autoencoder.

**Figure 7:** SAE architecture.

**Figure 8:** CT lung COVID-19 image cases that include normal and COVID-19 samples.

**Algorithm 1:** Deep learning-based COVID-19 diagnosis algorithm.

**Table 1:** CNN parameters.

Layer	Type	Input	Kernel	Output
1	Convolution layer	32 × 32 × 1	6 × 6	28 × 28 × 36
2	Max pooling	28 × 28 × 36	3 × 3	24 × 24 × 64
3	Convolution layer	24 × 24 × 64	6 × 6	20 × 20 × 64
4	Max pooling	20 × 20 × 64	3 × 3	12 × 12 × 64
5	Fully connected layer	12 × 12 × 64	5 × 5	8 × 8 × 64
6	Fully connected layer	8 × 8 × 64	2 × 2	2 × 1
7	Softmax layer	2 × 1 result	-	Identification output

**Table 2:** DNN parameters.

Layer	Type	Input	Output
1	Input layer	24 × 24 × 1	576 × 1
2	Fully connected layer	576 × 1	304 × 1
3	Fully connected layer	304 × 1	256 × 1
4	Fully connected layer	256 × 1	128 × 1
5	Fully connected layer	128 × 1	64 × 1
6	Softmax layer	2 × 1	Identification output

**Table 3:** SAE parameters.

Layer	Type	Input	Output
1	Input layer	24 × 24 × 1	576 × 1
2	Fully connected layer	576 × 1	304 × 1
3	Fully connected layer	304 × 1	256 × 1
4	Fully connected layer	256 × 1	128 × 1
5	Softmax layer	2 × 1	Identification output

**Table 4:** Deep learning model results.

Deep learning models	Accuracy (%)	Sensitivity (%)	Specificity (%)
CNN	88.30	87.65	87.97
DNN	86.23	84.41	86.77
SAE	86.75	85.62	87.84

**Table 5:** The comparison of the proposed models with the current state-of-the-art works in terms of testing time.

Approaches	Testing time (s)
Wang et al. (2020) [16]	10
Xu et al. (2020) [22]	30
Kassani et al. (2020) [44]	0.03
CNN	0.002
DNN	0.04
SAE	0.02

**Table 6:** Comparison with benchmarked studies on CT lung COVID-19 images.

Study/year	Dataset (samples no.)	Accuracy (%)	Sensitivity (%)	Specificity (%)
Zhao et al. [42](2020)	275 CT scans	84.7	N/A	N/A
Amyar et al. [45] (2020)	1044 CT collected from 3 datasets	86	94	79
He et al. [46] (2020)	349 CT scans	86	N/A	N/A
Our proposed (CNN)	746 chest CT scans	88.30	87.65	87.97
Our proposed (DNN)	746 chest CT scans	86.23	84.41	86.77
Our proposed (SAE)	746 chest CT scans	86.75	85.62	87.84

The article "Automated System for Identifying COVID-19 Infections in Computed Tomography Images Using Deep Learning Models" was retracted in 2023. Reasons: signs of a paper mill; suspected computer-generated content; unreliable results or conclusions; concerns about the data.

## Data Availability

The datasets generated during and/or analysed during the current study are available in the Barrett, J.F. and Keat, N., 2004. Artifacts in CT: recognition and avoidance. Radiographics, 24(6), pp.1679-1691.
